# Effects of Different Types of Early Restrictive Fluid Resuscitation on Immune Function and Multiorgan Damage on Hemorrhagic Shock Rat Model in a Hypothermic Environment

**DOI:** 10.1155/2022/4982047

**Published:** 2022-07-06

**Authors:** Linlin Xu, Lin Li, Jianyu Zu, Xinyuan Huang, Lin Tian, Yingjie Sun, Yugang Diao

**Affiliations:** ^1^Department of Anesthesia, Postgraduate Training Base of Jinzhou Medical University in the General Hospital of Northern Theater Command, Shenyang 110016, China; ^2^Department of Anesthesia, General Hospital of Northern Theater Command, Shenyang 110016, China; ^3^Department of Anesthesiology, Suzhou BOE Hospital 215505, China; ^4^Department of Anesthesia, General Hospital of Northern Theater Command, Shenyang, China

## Abstract

**Objective:**

This study was aimed at investigating the effects of different types of fluid restriction fluid resuscitation on the immune dysfunction and organ injury of hemorrhagic shock rats under a hypothermic environment.

**Methods:**

SD rats were divided into sham operation group (SHAM), hemorrhagic shock model group (HS), crystal liquid limited resuscitation group (CRLLR), colloidal liquid limited resuscitation group (COLLR), and nonlimited resuscitation group (NLR); rats in each group were placed in a low-temperature environment of 0-5°C for 30 min, and then, a hemorrhagic shock rat model was prepared. Sodium lactate Ringer's restricted resuscitation solution, hydroxyethyl starch restricted resuscitation solution, and hydroxyethyl starch were used for resuscitation, and hemodynamic examination was performed. The mortality rate, inflammatory factors, oxidative stress factors, and immune function were detected by ELISA. The dysfunction and injury of the intestinal, lung, liver, and kidney were examined by histological methods.

**Results:**

Hemorrhagic shock resulted in decreased immune function and activation of inflammation. Unrestricted fluid infusion further activated the inflammatory response. The crystalloid-restricted fluid infusion performed effectively to regulate inflammatory response, promote antioxidative activity, and reduce the immunosuppressive reaction. Rehydration could regulate the coagulation. The hydroxyethyl starch reduced the expression of platelet glycoproteins Ib and IIb/IIIa and blocked the binding of fibrinogen to activated platelets, thereby inhibiting intrinsic coagulation and platelet adhesion and aggregation. Rats in the CRLLR group showed to relieve the injury of the lung, liver, kidney, and intestine from hemorrhagic shock in low-temperature environment.

**Conclusion:**

The early application of restrictive crystalloid resuscitation in hemorrhagic shock rats in hypothermic environment showed the best therapy results. Early LR-restrictive fluid replacement promotes the balance of inflammatory response and the recovery of immunosuppressive state, resists oxidative stress, stabilizes the balance of coagulation and fibrinolysis, improves coagulation function, and relieves organ injury.

## 1. Introduction

Hemorrhagic shock (HS) is a syndrome caused by hypoperfusion of tissues and impairment of body organs and dysfunctions leading to blood loss exceeding 30% [1, 2]. Inadequate perfusion of tissues and organs stimulates the body to produce large amounts of inflammatory factors. It initiates systemic inflammatory response syndrome (SIRS), which eventually leads to multiple organ dysfunction (MODS) or even death if not treated promptly [3]. External factors such as high temperature, low temperature, plateau, and other extreme environments can exacerbate the body metabolism, energy consumption, and coagulation dysfunction [4]. As the prolonged time and tissue hypoxia result in multiorgan damage, it poses new challenges to late resuscitation, anesthesia, and perioperative management.

Deep hypothermia not only reduced the temperature of HS patients but is also correlated with the prognosis and survival rate of HS patients [5]. Once hypothermia occurs, the body increases the heat production, and oxygen consumption maintains the body temperature. The chilling response of the shocked body is suppressed, and heat production is reduced. As tissue oxygen consumption is limited by shock, hypothermia is further exacerbated by insufficient heat production. Early hypothermia increases the cardiac output and oxygen consumption, while later hypothermia can inhibit myocardial contractility and decrease the cardiac output [6]. It demonstrated that shock can trigger hypothermia and that spontaneous hypothermia due to hypothermic exposure can exacerbate hemorrhagic shock [7]. Therefore, the management of hemorrhagic shock in a hypothermic environment is very important.

Fluid resuscitation is the primary resuscitation measure for hemorrhagic shock [8]. The early studies suggested that massive and rapid fluid rehydration would be beneficial for patients in shock, restoring blood pressure and adequate perfusion of organs rapidly and promoting an improved prognosis [9]. However, the current studies suggest that massive and rapid rehydration may interfere with the body compensatory mechanisms for blood loss in shock, which may cause coagulation dysfunction, metabolic acidosis, and deterioration in the body internal environment, thereby increasing mortality [10]. Meanwhile, increasing blood flow, promotion of perfusion pressure, and reduction of blood viscosity may cause the destruction of preexisting blood clots and cause secondary bleeding. It has been shown that before bleeding in hemorrhagic shock, the controlling of obtaining minimal perfusion pressure could effectively reduce the blood loss and increase patient survival [11]. It has been shown that restrictive fluid resuscitation can be effective in using the body compensatory mechanisms to fully exploit the effects of fluid resuscitation and maintain mean arterial pressure (MAP) at approximately 50 mm Hg, i.e., improving tissue perfusion and animal survival [12]. There is a close relationship between the imbalance of proinflammatory and anti-inflammatory and shock development, and the rational regulation of inflammatory factors to reduce their damage to the organism was focused on by many researchers [13]. In this study, we established the HS rat model in a hypothermic environment, and we performed restrictive fluid resuscitation on HS rats using different fluid resuscitation methods to investigate the effects of restrictive fluid resuscitation on the immune function of rats in hemorrhagic shock, as well as to observe the impact on individual organ damage.

## 2. Materials and Methods

### 2.1. Laboratory Animals and Grouping

Specific pathogen-free, eight-week-old, male, Sprague Dawley (SD) rats were purchased from Liaoning Changsheng Biotechnology Co., Ltd. (SCXK (Liao) 2020-0001). The whole animal experiments were performed in the animal facility of the Department of Laboratory Animals, China Medical University. The whole animal experiment was approved by the Ethics Committee of Laboratory Animal Welfare of China Medical University (Approved No. CMU2020198). The rats were divided into sham-operated group (SHAM), hemorrhagic shock model group (HS), crystal liquid limited resuscitation group (CRLLR), colloidal liquid limited resuscitation group (COLLR), and nonlimited resuscitation group (NLR), with 20 rats in each group, using the random number table method.

### 2.2. Establishment of a Rat Model of Hemorrhagic Shock in a Hypothermic Environment

The rats in each group were anesthetized by intraperitoneal injection of sodium pentobarbital (35 mg/Kg, Sigma), the left carotid artery was cannulated in the supine position, and the right femoral artery was cannulated, and the rats' heart rates (HR), systolic blood pressure (SBP), diastolic blood pressure (DBP), and mean arterial pressure (MAP) were automatically collected and recorded. The left femoral vein was isolated, cannulated, and secured for rehydration, and 0.3% heparin saline (1 ml/kg) was administrated for rehydration after shock resuscitation. The rats were placed in a low-temperature environment at 0-5°C and stabilized for 30 min before bleeding starts. The first bleeding rate was 20 ml/kg at an interval of 5 min, and the second bleeding rate was 5 ml/kg. The MAP of rats was reduced to 40 mm Hg within 10 min and maintained at this blood pressure level for 30 min.

In the SHAM group, rats were not bleeding and not rehydrated, only the same surgical procedure. In HS group, rats were established for the shock model and maintained for 1 h, and rats were not resuscitated with any medicine and died of natural causes. In the CRLLR group (crystal liquid limited resuscitation group) and CRLLR (crystal liquid limited resuscitation group), 1 h after arterial cannulation and shock model establishment, 20 ml of sodium lactate Ringer's restricted resuscitation solution was administered to maintain MAP at 50 mm Hg. In the COLLR (colloidal liquid limited resuscitation group), 1 h after HS model establishment, 20 ml of hydroxyethyl starch was administered to maintain MAP at 50 mm Hg. In the nonlimited resuscitation group (NLR), 40 ml of hydroxyethyl starch was infused 1 h after the HS model was established, and the MAP was maintained at 80 mm Hg for 10 min before ending the infusion. The infusion was stopped after maintaining the MAP at 80 mm Hg for 10 min. The mortality rates in each group were observed within 6 h after the cessation of rehydration.

### 2.3. Hemodynamic, Coagulation, and Liver and Kidney Function Monitoring

The heart rate (HR) and mean arterial pressure (MAP) of rats were recorded before bleeding (T0), one hour after shock (T1), and one hour after resuscitation (T2), respectively; the femoral venous blood of each group was collected for testing the TEG indicators at each time point, including *R* value, *K* value, *α* angle, maximum thrombus amplitude (MA) value, coagulation index (CI) value, and half-hour fibrinolysis rate (LY30). The blood of each group of rats was collected after 6 h of HS for the detection of BUN, creatinine (Cr), ALT, and AST.

### 2.4. ELISA Assay

After six hours HS treatment, plasma was separated from the blood of rats, and the levels of inflammatory factors (TNF-*α*, IL-6, IL-8, and IL-10) and oxidative stress factors (malondialdehyde (MDA) and glutathione (GSH)) were measured by ELISA kits. The procedure was carried out according to the instructions.

### 2.5. Flow Cytometry

After six hours of HS treatment, lymphocytes were isolated from the blood of rats, incubated with CD^3+^, CD^4+^, and CD^8+^ antibodies for 30 min, washed with PBS, and detected by flow cytometry on the machine for content of CD^3+^CD^4+^ cells and CD^3+^CD^8+^ cells. The percentage of CD^3+^CD^4+^ plus CD^3+^CD^8+^ cells was also calculated.

### 2.6. Pathological Histological Examination

After six hours of HS treatment, rats' liver, kidney, lung, and intestinal tissues were fixed in neutral formalin for 48 h and rinsed in ddH_2_O. Then, tissues were dehydrated in gradient alcohol at 70%, 80%, 90%, 95%, and 100%, transparent in xylene, immersed in wax for 3 h. Paraffin-embedded wax was blocked; slices were cut into 5 *μ*m sections. After oven at 37°C overnight, the slices were dewaxed. The sections were stained with hematoxylin-eosin and sealed with neutral gum, and the histomorphology was observed under light microscopy. The lung tissues of rats were collected, weighed, and then dried in an oven at 80°C for 24 h to reach a constant weight. Formula: lung (intestine) water content = (wet weight − dry weight)/wet weight × 100%.

### 2.7. Western Blot Assay

Tissues were collected, homogenized, and added with lysis solution RIPA (Thermo, 89900) containing protease inhibitors on ice for 30 min; the supernatant of lysis protein was collected. Then, the concentration of lysis protein was quantified by BCA kit (Thermo Fisher Scientific, Inc.). The same amount of protein was loaded and separated with SDS-PAGE and transferred to a PVDF membrane. After being blocked in silk milk solution, the PVDF membrane was incubated with diluted anti-I-FABP antibody or anti-GAPDH antibody incubating overnight at 4°C; PVDF membranes were washed with PBS. Then, HRP-conjugated secondary antibodies were added and incubated at room temperature for 2 h. Proteins were visualized using the ECL luminescence kit and gel imaging system. Finally, blots were analyzed using ImageJ software.

### 2.8. Statistical Analysis

Statistical analysis was performed using SPSS 22.0, and results were expressed as mean ± standard deviation (S.D.). The group comparisons were performed by student *t* test. One-way ANOVA was used for multiple group comparisons; *P* < 0.05 was considered as a statistically significant difference.

## 3. Results

### 3.1. The Regulatory Effect on Hemodynamic Changes and Coagulation Function by Early Restrictive Fluid Resuscitation

Firstly, we successfully prepared the HS rat model. The survival percentage of rats in different groups was 100% in the SHAM group, 20% (4 rats) in the HS group, 65% (13 rats) in the CRLLR group, 45% (9 rats) in the COLLR group, and 30% (6 rats) in the NLR group (Figure 1(a)). HR and MAP values were also monitored to demonstrate the hemodynamic changes. The results showed that there was no significant difference in HR between the groups before bleeding (T0) (*P* > 0.05), and there was no significant difference between the groups at 1 h after bleeding (T1) compared to T0 (*P* < 0.05). The HR of rats in each group increased compared to T1 at 1 h after resuscitation (T2). The HR of rats in the CRLLR group was lower than that of the COLLR group, and the HR of both groups was higher than that of the SHAM group. The heart rates in the NLR group were a little more than that in the CRLLR and COLLR groups. The heart rates in the NLR group were much more than that in the HS group (Figure 1(b), *P* < 0.05).

The MAP of the rats in each group was not significantly different before bleeding (T0) (Figure 1(c), *P* > 0.05), and the MAP of the rats in each group decreased significantly at one hour after bleeding (T1) compared to T0 (*P* < 0.01), and there was no significant difference between the groups (*P* > 0.05). The MAP of rats in the CRLLR group was higher than that of the COLLR group and lower than that of the SHAM group, and that of the NLR group was lower than that of the two groups with restricted rehydration, however higher than that of the HS group one hour after resuscitation (T2) (Figure 1(c), *P* < 0.05).

### 3.2. The Regulatory Effect on Coagulation Function by Early Restrictive Fluid Resuscitation

Coagulation dysfunction is one of the difficulties in the rescue of hypothermic HS and an important factor in the survival rate of HS rescue, which includes hyperfibrinolysis and platelet dysfunction. We assessed the coagulation function of rats at each time point by thromboelastography, and *R* value (Figure 2(a)) responded to the function of coagulation factors and *K* value (Figure 2(b)) responded to the number and function of platelets, and the results showed that the *R* value of each group of rats at T1 was higher than that of T0 (*P* < 0.05), and there was no statistical significance among the groups. *R* values of rats in the rehydration group were promoted, which is the highest in the unrestricted rehydration group, followed by the HS group. The *R* value of rats in the CRLLR group was lower than those in the COLLR group in the restricted rehydration group (*P* < 0.05), and *K* values and *R* values of rats in all groups at the three time points were consistent. The *α* angle (Figure 2(c)), MA values (Figure 2(d)), and CI values (Figure 2(e)) of rats in all groups at T1 were lower than those at T0 (*P* < 0.05), and there was no statistical significance between all groups at both time points. The *α* angle, MA values, and CI values of rats in all groups in hemorrhagic shock at T1 were lower than those in the SHAM group, and at T2, compared with the SHAM group, the *α* angle, MA values, and CI values of rats in the HS group and each rehydration group decreased, with the HS group being the lowest, followed by the unrestricted rehydration group, and the CRLLR group being higher than the COLLR group (*P* < 0.05); the LY30 of rats (Figure 2(f)) in all groups at T1 was higher than that at T0 (*P* < 0.05), which was not statistically significant among all groups. The LY30 of rats in each group of hemorrhagic shock was significantly higher at T1 compared with the SHAM group, and at T2 compared with the sham-operated group, the LY30 of rats in both the HS group and each rehydration group was higher, with the HS group being the highest, followed by the unrestricted rehydration group, and the LY30 of rats in the CRLLR group was lower than that of the COLLR group in the restricted rehydration group (*P* < 0.05). The above results indicate that unrestricted rehydration had the greatest effect on coagulation during resuscitation after hemorrhagic shock, and the short duration of heavy rehydration caused excessive blood dilution including imbalance of procoagulant and anticoagulant factors and dysfunctional cell swelling, resulting with deterioration of coagulation.

### 3.3. The Effect on Inflammatory Factors, Oxidative Stress Factors, and Immune Function of Rats under Different Fluid Resuscitation Treatment

In the end of the whole experiment, TNF-*α*, IL-6, IL-8, and IL-10 were significantly higher in the HS group compared with SHAM group, and TNF-*α*, IL-6, and IL-8 were higher in the NLR group than in the HS group in all groups of rehydrated rats (Figures 3(a)–3(c), *P* < 0.05). The content of TNF-*α*, IL-6, and IL-8 in restricted rehydration group was lower than that in the HS group, in which CRLLR group was lower than that in the COLLR group (Figures 3(a)–3(c), *P* < 0.05). The level of IL-10 was lower in the NLR group than that in the HS group and higher in the CRLLR group than that in the COLLR group; all groups were slightly greater than the HS group (*P* < 0.05). We further examined MDA and GSH levels in rats to assess the change in oxidative stress, and the results showed that MDA (Figure 3(e)) and GSH (Figure 3(f)) levels were higher in the HS group compared to that in the SHAM group, followed by the NLR group, and lower in the CRLLR group compared to the COLLR group (*P* < 0.05). CD^3+^CD^4+^ and CD^3+^CD^8+^ lymphocytes were significantly reduced in the HS group compared to that in the SHAM group. CD^3+^CD^4+^ and CD^3+^CD^8+^ (Figure 3(g)) lymphocytes in the NLR group were lower than the HS group, in which the CRLLR group was the highest, followed by the COLLR group. The above results showed that blood loss shock caused the body immune function to be inhibited and the inflammation was activated, and nonrestricted rehydration further activated the inflammatory response, while crystal-restricted rehydration was more advantageous in regulating the inflammatory response and antioxidative stress and reducing the immunosuppressed state of shock.

### 3.4. HS Relieved the Intestinal Injury

Moreover, the effect of intestinal fatty acid binding protein (I-FABP) assay, intestinal wet-to-dry ratio, small intestinal tissue HE, and the application of different doses of fluid resuscitation on intestinal injury in rats in hemorrhagic shock were also assessed. The results showed that I-FABP levels (Figures 4(a) and 4(b)) were significantly higher in the hemorrhagic shock group compared to that in the SHAM group, followed by the NLR group and lower in the CRLLR group than the COLLR group (*P* < 0.05). The intestinal wet-to-dry ratio (Figure 4(c)) was consistent with the I-FABP results. Restrictive crystalloid rehydration resuscitation had the least effect on intestinal mucosal injury after hemorrhagic shock.

### 3.5. HS Leads to Lung Injury

Hemorrhagic shock can cause acute lung injury, which can develop into acute respiratory distress syndrome in severe cases. The pathology of ALI is characterized by increased alveolar capillary permeability and lung tissue oedema. Therefore, we assessed the severity of vascular permeability and pulmonary oedema in rats by quantifying the wet/dry (W/D) ratio (Figure 5(a)) of the lungs, and the morphological damage of lung tissue was observed by HE staining (Figure 5(b)) and analyzed pathologically. The results showed that the lung W/D weight ratio was significantly higher in all groups of rats in hemorrhagic shock at 6 h in the HS compared with the SHAM group, with the highest lung W/D weight ratio in the HS group, followed by the NLR group, and a lower lung W/D weight ratio in the CRLLR group than in the COLLR group (*P* < 0.05). HE staining data of lung tissue were consistent with the above results. The lung tissues in the SHAM group showed clear structures of each bronchus, alveoli, and alveolar septum, with no obvious inflammatory cell infiltration and no abnormal manifestations such as hemorrhage, exudation, and oedema. The lung tissue of the rats in the hemorrhagic shock group showed disorganized structures, inflammatory cell infiltration, alveolar wall thickening, massive alveolar fusion, and pink exudate in the alveolar cavity, while the CRLLR group showed less intra-alveolar congestion and exudation and interstitial inflammatory cell infiltration (*P* < 0.05).

### 3.6. HS Results to the Liver and Kidney Dysfunction

The plasma urea and Cre levels were significantly higher in the HS group compared to the SHAM group, with the highest urea and creatinine levels in the HS group (Figures 6(a), *P* < 0.05). We observed histopathological changes in the kidneys (Figure 6(b)) showing normal histopathological sections with normal glomerular structure in the SHAM group under high magnification and oedema in the HS group. The glomerular structure was fragmented, the tubular epithelium was swollen, the lumen was narrowed, and the renal blood vessels were congested. The kidney tissue in the NLR group was mildly oedematous. The glomerular structure was mildly fragmented, a few tubular epithelial cells were swollen, and the renal vessels were mildly congested. The pathological phenotype in the COLLR groups was slightly recovered and better than those of the NLR group. The glomerular structure of these groups was basically normal, with scattered inflammatory cells and occasional congestion of the renal vessels. Our data suggest that hemorrhagic shock causes ALI. The restrictive rehydration resuscitation is less damage to the kidney, with no significant differences observed between crystalloid and colloid restrictive resuscitation methods.

The plasma ALT and AST were examined. The plasma ALT and AST were significantly increased in all groups of rats in HS 6-hour hemorrhagic shock compared to the SHAM group, and plasma ALT and AST were the highest level in rats of the HS group, decreased in the CRLLR group, and increased in the NLR group compared to the COLLR group, suggesting that restrictive colloidal rehydration was effective in improving hemorrhagic shock hepatic impairment after resuscitation. The results of the pathological changes observed showed that rats in the SHAM group was essentially uninjured as that in the control group. The liver tissue injury was more severe in the SH group, followed by the NLR group. The injury in the CRLLR group was less severe than that in the COLLR group (Figure 6(c), *P* < 0.05).

## 4. Discussion

The fluid resuscitation is one of effective treatments of hemorrhagic shock in a hypothermic environment [14]. In this study, we investigated the effects of different resuscitation methods and different resuscitation fluids on immune function and organ damage after resuscitation of rats in posttraumatic hemorrhagic shock. The results showed that rats resuscitated with crystal-restricted rehydration fluids caused the least inflammatory immune system disorders and organ damage after hemorrhagic shock. The effective fluid resuscitation after hypothermic hemorrhagic shock is important in restoring the body circulating blood volume, ensuring circulatory perfusion of tissues and organs and delaying the progression of shock. Recently, the early restrictive fluid resuscitation has been recommended for maintaining the microcirculatory perfusion, reducing blood loss, mitigating inflammatory responses, adjusting internal environmental stability, and reducing ischaemia-reperfusion injury [15]. A meta-analysis investigation on nine animal found the reduced mortality after hemorrhage in animals receiving hypotensive fluid resuscitation compared to those receiving normotensive resuscitation [16]. Our study demonstrated that early application of crystal-restricted rehydration resuscitation in a hypothermic environment was effective in stabilizing circulation and improving survival in rats in hemorrhagic shock. We observed that the early nonrestricted entry of large amounts of fluid into the bloodstream caused dilution of coagulation factors and reduced platelet function, resulting in further deterioration of coagulation and that the application of LR rehydration fluids during restrictive resuscitation had a lower effect on coagulation than HES. The hydroxyethyl starch could inactivate or degrade the coagulation factor V, factor VIII, and von Willebrand factor through combination [17]. In addition, hydroxyethyl starch reduces the expression of platelet glycoproteins Ib and IIb/IIIa and inhibits the binding of fibrinogen and activated platelets, thereby inhibiting endogenous coagulation and platelet adhesion and aggregation [17]. Other studies have demonstrated that hydroxyethyl starch can inhibit platelet function and increase bleeding tendency by blocking ligand binding to surface receptors and nonspecific modification of cell membrane structure [18]. These studies supported that the early crystal-restricted rehydration attenuated the coagulation disorders after resuscitation from hypothermic hemorrhagic shock.

Shock is closely related to immunity, which could activate the body immune system, leading to an excessive inflammatory response [19]. The abnormal inflammatory state causes the body immune system to damage endothelial tissues and ultimately organs, in addition to the postischaemic reperfusion injury of shock, which further activates neutrophils and mediates the release of cytokines and free radicals probably leading to secondary damage. The early and rapid fluid resuscitation was reported to lead to immune damage and exacerbates the inflammatory response [20]. In this study, we showed that the inflammatory response is activated in the early phase of hemorrhagic shock in a hypothermic environment, and the inflammatory factors including TNF-*α*, IL-6, IL-8, and IL-10 are significantly increased, and the plasma proinflammatory factors such as TNF-*α*, IL-6, and IL-8 are increased, while the levels of anti-inflammatory factor IL-10 are decreased in rats given unrestricted fluid resuscitation. LR-restricted rehydration was more effective in inhibiting proinflammatory factors and promoting anti-inflammatory effects, while restricted rehydration was effective in antioxidation, and the levels of MDA and GSH in rats in the NLR group were significantly higher than those in the restricted rehydration group. We measured CD^3+^CD^4+^ and CD^3+^CD^8+^ lymphocytes using flow cytometry, and the crystal-restricted rehydration group was higher than the colloid-restricted rehydration group. Both groups were higher than the nonrestricted rehydration group. These results suggest that early crystal-restricted rehydration restores the dynamic balance of proinflammatory and anti-inflammatory factors in the body, reduces the level of inflammatory factors, effectively counteracts oxidative stress, and improves the immunosuppression caused by shock. It has been reported that HES stimulates the formation of platelet neutrophil couples to exert a proinflammatory effect [21]. LR contains electrolytes similar to plasma and is effective in avoiding hyperchloremic acidosis, which has been shown to be associated with a proinflammatory immune response, during rehydration [22]. Schultz et al. have reported that early resuscitation using lactated Ringer's solution could reduce gut ischaemia and promote the function of gut barrier to inhibit the inflammatory response [23].

Ischaemia-reperfusion injury in hemorrhagic shock, coagulation dysfunction, and inflammatory responses ultimately leads to multiple organ dysfunction [24–26]. We examined histopathological changes, biochemical parameters, and several molecule biomarkers to investigate the effects of different fluid resuscitation modalities on organ function in rats in hemorrhagic shock. In the nonrestricted fluid resuscitation group, the rats perform less oedema, necrosis, and inflammatory cell infiltration in the small intestine, lung, liver, and kidney, while the restricted fluid resuscitation group had significantly less histopathological damage in all organs and lower wet/dry weight ratios and biochemical parameters in intestinal and lung tissues. The early stage of hemorrhagic shock significantly reduced intestinal blood perfusion and disrupted intestinal mucosal barrier function, leading to systemic inflammatory responses induced by translocation of bacteria or endotoxins. Meanwhile, the ischaemia-reperfusion damage caused by hemorrhagic shock further activates the inflammatory response, leading to tissue oedema, exudation, and even necrosis. Several animal and clinical trials have confirmed that the key factors in organ damage after hemorrhagic shock is the inflammatory response [27–29]. Our results demonstrate that crystal-restricted rehydration is better at restoring inflammatory homeostasis, counteracting oxidative stress, and promoting recovery from immunosuppression. Early rapid and massive fluid replacement causes excessive haemodilution, exacerbating hypoxia and coagulation dysfunction, while high intravascular hydrostatic pressure exacerbates endothelial damage and cellular swelling dysfunction. Restrictive rehydration is effective in stabilizing circulation, restoring tissue perfusion, and avoiding the damage caused by rapid and massive rehydration. Early application of LR-restrictive rehydration fluid is helpful in restoring the intracellular environment and reducing ischaemia-reperfusion injury. In contrast to HES, it also reduces the viscosity of the blood, unblocks the microcirculation, and facilitates oxygen delivery and cytokine metabolism, thus improving organ function. Colloids are large in molecular weight, which are effective in maintaining the simplified osmotic pressure of plasma [30]. Colloids hardly get through cell membranes, leading to dehydration of red blood cells, and early colloidal rehydration aggravates tissue hypoxia and affects coagulation [31]. Some studies have suggested that colloid-restricted rehydration is superior to crystalloid-restricted rehydration [32]. In this study, we detected the rat model living for 24 hours after resuscitation in a noncold environment for 30 min. Early restrictive crystalloid resuscitation has a transient hemodynamic beneficial effect, and because crystals tend to leak out of the tissue spaces, continued application of crystalloid rehydration at a later stage increases tissue oedema and affects tissue oxygenation, exacerbating tissue damage [33]. Our study used hemorrhagic shock rats with either LR or HES for rehydration resuscitation, which does not fully simulate clinical resuscitation protocols. However, this study could provide more clinically relevant fluid resuscitation protocols to explore the effects of different fluid resuscitations for hypothermic hemorrhagic shock on the organism to assist in clinical resuscitation efforts.

## Figures and Tables

**Figure 1:** Early restrictive fluid resuscitation regulates hemodynamic changes and coagulation function of HS rat model. (a) The percentage of survival rate of rats in different groups. (b) The times of mice heart rates in different groups. ns, *P* > 0.05; ∗, *P* < 0.05 vs. same group at T0; #, *P* < 0.05 vs. NLR at T2. (c) The MAP value of mice in different groups. ns, *P* > 0.05; ∗, *P* < 0.05 vs. same group at T0; $, *P* < 0.05 vs. COLLR at T2; #, *P* < 0.05 vs. NLR. SHAM: sham-operated group; HS: hemorrhagic shock model group; CRLLR: crystal liquid limited resuscitation group (CRLLR); COLLR: colloidal liquid limited resuscitation group; NLR: nonlimited resuscitation group.

**Figure 2:** The regulatory effect on coagulation function by early restrictive fluid resuscitation. (a) The *R* values of rats in different time points. (b) The *K* values of rats in different time points. (c) The *α* angle values of rats in different time points. (d) The MA values of rats in different time points. (e) The CI values of rats in different time points. (f) The LY30 values of rats in different time points; ns, *P* > 0.05; $, *P* < 0.05; #, *P* < 0.05 vs. COLLR at same time point; ∗, *P* < 0.05 vs. SHAM at same time point; SHAM: sham-operated group; HS: hemorrhagic shock model group; CRLLR: crystal liquid limited resuscitation group (CRLLR); COLLR: colloidal liquid limited resuscitation group; NLR: nonlimited resuscitation group.

**Figure 3:** The effect on inflammatory factors, oxidative stress factors, and immune function of rats under different fluid resuscitation treatment. (a) The concentration of TNF-*α* of rats in different groups. (b) The level of IL-6 of rats in different groups. (c) The concentration of IL-4 of rats in different groups. (d) The concentration of IL-10 of rats in different groups. (e) The concentration of MDA of rats in different groups. (f) The level of GSH of rats in different groups. ns, *P* > 0.05; $, *P* < 0.05; ∗, *P* < 0.05 vs. SHAM at same time point; #, *P* < 0.05 vs. COLLR at same time point. SHAM: sham-operated group; HS: hemorrhagic shock model group; CRLLR: crystal liquid limited resuscitation group (CRLLR); COLLR: colloidal liquid limited resuscitation group; NLR: nonlimited resuscitation group.

**Figure 4:** HS relieved the intestinal injury. (a) Western blot results of I-FABP. (b) The relative gray value of western blot results. (c) The ratio of wet to dry weight in rats' intestinal of different groups. ∗, *P* < 0.05 vs. SHAM; $, *P* < 0.05; #, *P* < 0.05 vs. COLLR. SHAM: sham-operated group; HS: hemorrhagic shock model group; CRLLR: crystal liquid limited resuscitation group (CRLLR); COLLR: colloidal liquid limited resuscitation group; NLR: nonlimited resuscitation group.

**Figure 5:** The lung injury resulted by HS treatment. (a) The ratio of dry to wet lung weight. ∗, *P* < 0.05 vs. SHAM; $, *P* < 0.05; #, *P* < 0.05 vs. COLLR. (b) The HE staining results of rats' lung tissue. Scale bar = 5 *μ*m. SHAM: sham-operated group; HS: hemorrhagic shock model group; CRLLR: crystal liquid limited resuscitation group (CRLLR); COLLR: colloidal liquid limited resuscitation group; NLR: nonlimited resuscitation group.

**Figure 6:** The effect of liver and kidney dysfunction under HS treatment. (a) The levels of BUN and Cre in rat plasma of different groups. ∗, *P* < 0.05 vs. SHAM; $, *P* < 0.05; #, *P* < 0.05 vs. HS. (b) HE staining results in the rats' kidney. Scale bar = 5 *μ*m. (c) The levels of ALT and AST in the rats' plasma. ∗, *P* < 0.05 vs. SHAM; $, *P* < 0.05; #, *P* < 0.05 vs. COLLR. SHAM: sham-operated group; HS: hemorrhagic shock model group; CRLLR: crystal liquid limited resuscitation group (CRLLR); COLLR: colloidal liquid limited resuscitation group; NLR: nonlimited resuscitation group.

## Data Availability

No data were used to support this study.
